# Evaluation of Antimicrobial and Wound Healing Effects of Gold Nanoparticles Containing *Abelmoschus esculentus* (L.) Aqueous Extract

**DOI:** 10.1155/2021/7019130

**Published:** 2021-10-22

**Authors:** Shahla Korani, Khodabakhsh Rashidi, Mona Hamelian, Ali R. Jalalvand, Ahmad Tajehmiri, Mitra Korani, Thozhukat Sathyapalan, Amirhossein Sahebkar

**Affiliations:** ^1^Research Center of Oils and Fats, Kermanshah University of Medical Sciences, Kermanshah, Iran; ^2^Academic Diabetes Endocrinology and Metabolism, Hull York Medical School, University of Hull, United Kingdom of Great Britain and Northern Ireland, Hull, UK; ^3^Applied Biomedical Research Center, Mashhad University of Medical Sciences, Mashhad, Iran; ^4^Biotechnology Research Center, Pharmaceutical Technology Institute, Mashhad University of Medical Sciences, Mashhad, Iran; ^5^School of Pharmacy, Mashhad University of Medical Sciences, Mashhad, Iran

## Abstract

*Background*. Wound healing is a complex process of replacing devitalized cellular structures and tissues with healthy cells and tissue. Nanotechnology has been increasingly proposed as a novel platform to treat wounds and skin regeneration. The aim of this study was to evaluate the antibacterial, antioxidant, cytotoxic, and cutaneous wound healing activities of phytosynthesized Au NPs using *Abelmoschus esculentus* (okra) and synthesized Au NPs by using the citrate synthesis method. The Ok Au NPs were characterized using various techniques like UV-Vis absorption spectroscopy, FTIR, X-ray diffraction (XRD), and transmission electron microscopy (TEM). Cutaneous wounds were created on 30 rats and randomized into three groups: untreated and two groups treated with Ch Au NPs and Ok Au NPs. The treatment was carried out daily for 12 days. A peak characterized the Ok Au NPs at 538 nm in the UV-Vis spectrum. Based on the results of FTIR spectroscopy, various functional oxygenated groups such as hydroxyl, carboxyl, and nitrogenous groups were observed. XRD confirmed the crystalline nature of the nanoparticles. TEM images of Ok Au NPs showed a spherical shape and size range of 75 nm. DPPH test showed similar antioxidant potentials for Au NPs. The Au NPs showed cell viability in a dose-dependent manner, and this technique was found to be nontoxic. Agar well diffusion, which is the method to determine antibacterial characteristics of Au NPs, showed a significant beneficial effect against a variety of bacterial species. In addition, histopathological results showed that Au NPs could accelerate wound closure. Therefore, Au NPs could be suitable for wound healing applications.

## 1. Introduction

The skin is the largest organ in our body and acts as the first effective defense against the outside environment. The skin protects the body from exogenous organisms and substances. When a wound occurs to the skin, a series of active events begin rapidly, resulting in significant changes in the immune system [1–3]. Therefore, one of the most crucial characteristics of an ideal wound dressing is disinfecting skin from exogenous organisms. Over the past 20 years, various new wound dressings loaded with antimicrobial drugs have been developed. These advanced dressings could actively eliminate the pathogens in the infected wounds, decrease bacterial bioburden, and inhibit reinfection during healing and surgical dressings. It is essential to mention that high microbial load leads to a considerable delay in wound healing and bacterial biofilm development is one of the crucial mediators in chronic wounds [4].

In recent years, a lot of attention has been paid to nanoscience and nanotechnology. Nanotechnology is concerned with nanoscale visualization, handling, and manufacture of substances [5]. Nanoparticles with different sizes, shapes, and chemical compositions have various ranges of applications [6]. A variety of methods, including physical (pulsed wire, pulse laser ablation, ball milling method, mechanical chemical synthesis, and mechanical/high ball milling technique), chemical (microemulsion/colloidal technique, chemical reduction technique, electrochemical method, solvothermal decomposition, and sonochemical technique), and biological techniques (plant extract, bacteria, fungi, and yeast) have been used in synthesis nanoparticles [7, 8].

In most of the physical techniques used for synthesizing nanoparticles, empirical factors are controlled in the presence of a reducing agent to regulate the nanoparticle composition and characteristics without contamination. The chemical reduction of metal ions in solutions is the easiest and commonest method used for their synthesis [9]. The application of physical techniques needs high cost, pressure, and temperature. On the other hand, most chemical techniques utilize toxic and dangerous chemicals that harm the biological systems and environment. The production of toxic products is another problem with the use of the chemical technique. Therefore, it seems necessary to find a very effective and cheap technique without toxins and environmental harm [7].

Owing to its simplicity, nontoxicity, and cost-effectiveness, the biological method is considered the best technique for synthesizing nanoparticles [10]. The compounds in the plant extract, such as phytochemicals, e.g., flavonoids, phenolics, vitamins, amino acids, and polysaccharides as reducing agents, could form nanoparticles. Nanoparticles that are synthesized by herbal extracts do not produce harmful chemicals. Therefore, they can be employed in medicine extensively [11, 12]. Nanotechnology by the function of nanomaterials opened a novel stage in wound healing treatment suggesting solutions to increase the speed of wound healing [13]. Two main nanoparticles are generally used in wound healing: nanoparticles that possess essential characteristics helping wound closure and nanoparticles employed as delivery routes for therapeutic agents. The first type can be divided into metallic nanomaterials and nonmetallic nanomaterials [14]. Metal-based nanomaterials are currently generating more interest by scientists for nanomedicine applications such as diagnosis and imaging, drug delivery, photodynamic therapy, and tissue engineering, due to structural properties, their size and shape, and their antioxidant functions [15–18].

Gold nanoparticles (Au NPs) have been investigated for medical applications such as wound healing because of their chemical properties, optical stability, and ease of surface modifications. For gold nanoparticles, fusion or surface modification with other biomolecules is needed before wound healing applications. For example, adding polysaccharide peptides to Au NPs enhances their potency to improve healing [19].

Gold nanoparticles act as antioxidants by inhibiting free radicals such as hydroxyl, nitric oxide, and hydrogen peroxide [20]. Gold nanoparticle application on cutaneous wounds increased the angiopoietin, VEGF, and collagen expressions and reduced MMP and TGF-*β*1 levels [21]. Gold nanoparticles have been applied in cancer therapy, biosensing, gene, drug delivery, imaging, and biocompatibility [22]. Besides, antibiotic-coated gold nanoparticles doped PCL/gelatin nanofiber mat was examined on infected full-thickness wounds. It exhibited reduced bacterial load and promoted healing [23].

Nanoparticles can be applied for the treatment of wound infections due to their unique properties. Therefore, researchers have tried to discover an alternative therapeutic method using safer green options such as plants. The synthesis of plant-based nanoparticles is stable, fast, and economical. Furthermore, these nanoparticles can be synthesized with diverse shapes and sizes [24].

*Abelmoschus esculentus* (L.) (okra) belongs to the *Malvaceae* family, a flowering plant. It is a herbal medicine used to treat wound healing with various advantageous properties, including antioxidant, antibacterial, antidiabetic, antiplasmodial, analgesic, anticancer, antidiarrheal, and anti-inflammation properties [25]. The okra fruit has chemical ingredients, including saponin, tannin, alkaloid, and flavonoid. Moreover, okra fruit has quercetin, which acts as an antioxidant and an antitumor agent. Its antioxidant properties are through inhibition of the migration of the endothelial cells [26]. Saponin is another active agent in okra fruit, exerting antibacterial activities and also stimulating angiogenesis. Furthermore, it was demonstrated that flavonoid, the mediator of collagen type III synthesis, acts as an anti-inflammatory agent, modulates the oxidative burst in neutrophils, and acts as a phospholipase inhibitor [27]. Flavonoids also decrease the reactive oxygen species (ROS). Therefore, it can potentiate wound healing [28]. In this study, we aimed to synthesize and characterize Au NPs using okra extract and demonstrate the cutaneous wound healing effects of Au NPs (Figure 1). To the best of our knowledge, there are no reports on applying the green OK Au NPs to wound healing purposes which is the novelty of this work.

## 2. Experimental Section

### 2.1. Materials

Phosphate buffer solution (PBS), Dulbecco's modified Eagle's medium (DMEM), penicillin-streptomycin solution, fetal bovine serum, dimethyl sulfoxide (DMSO), and 2, 2 diphenyl-1-picrylhydrazyl (DPPH) were obtained from Sigma-Aldrich (New York, USA) in analytical grade with maximum purity. Fresh *A. esculentus* fruit was obtained from the mountain of Kermanshah province (west of Iran).

#### 2.1.1. Preparation of Plant Extract

Fresh okra was washed 3 times with deionized water, dried at 30°C in the oven, and powdered by a mortar, and then 1 g of obtained powder was boiled in 200 mL of water for 20 min until the solution color changed to light yellow. The extract was filtered through Whatman filter no. 1.

#### 2.1.2. Biosynthesis of Gold Nanoparticles

For a typical experiment, freshly okra extract (5 mL) was mixed with an aqueous solution of (1 mM) HAuCl_4_ × H_2_O (95 mL) at room temperature. The light violet color appeared for 5 minutes, indicating the formation of Au NPs. The solution was stirred for 1 h, centrifuged at 12000 rpm for 10 min, and removed from the upper phase to complete the reduction process. The obtained Ok Au NPs were washed three times with deionized water. They were then dried in an oven at 50 °C.

#### 2.1.3. Chemical Synthesis of Gold Nanoparticles

Ch Au NPs were synthesized through 5 steps. (1) Aqua (3HCl : 1HNO_3_) was freshly prepared in a beaker under a hood. Magnetic stir bar, 200 ml two-neck flask, stopper, and condenser were soaked in aqua for 15 min. Then, the glassware was washed with deionized water 3 times. (2) HAuCl_4_ solution, 2 ml of 50 mM, was added to 98 ml of Millipore water into the two-neck flask. (3) The condenser was connected to one neck of the flask, the stopper was placed in the other neck, and the flask was put on the hot plate to reflux while stirring. (4) As the refluxing was initiated, the stopper was removed, immediately 10 ml of 38.8 mM sodium citrate was added, and the stopper was replaced. The color changed from yellow to dark red in 1 min. The system was refluxed for 20 min and again for 5 min [29].

### 2.2. Antioxidant Assay

#### 2.2.1. Measurement of Antioxidant Properties of Au NPs by DPPH

To determine the trapping potential of 1, 1 diphenyl-2-picrylhydrazyl (DPPH), different concentrations of Au NPs were prepared using an aqueous extract of okra and sodium citrate was mixed with 3 mL 0.004 DPPH solution. The control solution contained 1 mL DPPH and 3 mL methanol. The obtained solutions were shaken and then kept in the dark at room temperature for 30 min. Finally, the absorption rate of each sample was measured at 517 nm. All tests were done in triplicate. Ascorbic acid was used as the standard antioxidant. In addition, the percentage of DPPH scavenging activity was evaluated [30].

### 2.3. Evaluation of Cytotoxicity Assay

#### 2.3.1. Cell Cultures

HDF cell lines were obtained from the Pasture Institute of Tehran (Iran). Cell lines were cultured in DMEM and supplemented with 10% FBS and 1% penicillin-streptomycin [31].

#### 2.3.2. MTT Assay

The effect of Au NPs on cell viability was measured using the MTT (3-(4, 5-dimethylthiazol-2-yl)-2, 5-diphenyltetrazolium bromide) assay [32]. At 80% confluency, cells were exposed with different concentrations of Au NPs (0, 7.5, 15, 30, 60, 100, 150, and 200 *μ*g/mL) for 24 h. Then, 20 *μ*L/well MTT (5 mg/mL) was added to each well and was incubated at 37 °C for 4 h. Finally, 100 *μ*L of DMSO was added to the wells. The absorbance at 570 nm was measured with an ELISA reader.

### 2.4. Antimicrobial Activity

The MIC test was performed on a sterile 96-cell plate using the CLSI standard microdilution method and European Committee on Antimicrobial Susceptibility Testing (EUCAST). For evaluating the antibacterial activity, the four bacterial species *Escherichia coli* ATCC 11775*, Klebsiella pneumoniae* ATCC 13883 (Gram-negative bacterium), *Staphylococcus aureus* ATCC 33591*, and Bacillus subtilis* ATCC 6051 were purchased from the Persian Type Culture Collection. The culture medium alone and medium containing bacteria without tested compounds were used as controls. Bacterial culture was performed under aerobic conditions at 37 °C in a brain-heart infusion medium supplemented with fetal bovine serum (FBS 2 mL/litre) purchased from Sigma, UK. For each experiment, bacteria were grown in aerobic conditions as previously described [33]. Chloramphenicol and tetracycline with a concentration of 30 µg/ml were used as controls. The templets were weighed to 0.35 mg. Antibacterial effects of the mentioned extracts were compared with chloramphenicol and tetracycline. The bacterial cell suspension was adjusted to a turbidity of 0.5 McFarland standard (turbidity = McFarland barium sulfate standard 0.5). A concentration of 5 mg/ml MTT was prepared in PBS (pH 7.2) purchased from Sigma and used for the bacterial growth tests (indicator solution concentrations) [34]. Twenty *μ*l of MTT solution was added to every single well, and the 96-well microtiter plates were incubated for 30 min at 28°C. To avoid loss of formed formazan granules, 80% of the MTT solution was carefully removed. The insoluble purple formazan granules were solubilized with MTT lysis buffer (0.5% sodium dodecyl sulfate, 36 mM HCl, and isopropanol acid), and the absorbance was measured at 540 nm. To optimize the incubation time of the bacterial suspension with MTT solution, several incubation times (15 and 30 min) were tested. The ultimate absorbance for each well was calculated as follows: Ab (540 nm) of the sample − Ab (540 nm) of the control.

### 2.5. Well Diffusion Method

In another method, by creating a well on the culture medium by sterile pipette (with pipette number 5 and depth 4 mm), the bacterial suspension with a concentration equivalent to half McFarland was spread on the surface of the culture medium with a swap. All MIC and MBC analyses were performed in 2 replications. SPSS software (version 20) was used to analyze the data, and one-way analysis of variance (ANOVA) was used to analyze the differences between different treatments. The statistical analysis results showed a significant level for the studied nanoparticles (*p* < 0.05), and therefore, the studied nanoparticles had a lethal effect on microorganisms. The following equation was used to measure growth inhibition values (the results were expressed as mean ± SD) [35]: growth inhibition = (control OD − sample OD)/control OD × 100.

### 2.6. In Vivo Studies

Adult male *Sprague Dawley* rats (*n* = 30, weight: 200–250 g) were used to assess the position of wound healing. All experiments were performed according to the Animal Care and Use Protocol of Kermanshah University of Medical Sciences (Iran) and approved by the Ethical Committee of the Kermanshah University of Medical Sciences (approval no. 443).

Based on the Helsinki Protocol (Helsinki, Finland, 1975). The rats were kept in separate cages at 20 ± 2 °C with a 12 h/12 h light/dark cycle and free access to food and water. The animals were anesthetized by intramuscular administration of 50 mg/kg i.p. body weight of ketamine. After anaesthesia induction, the animals' back hair was shaven using an electronic shaver, and the exposed skin was washed with 70% ethanol. A full-thickness skin excision wound was made (2 cm in diameter). After creating the cutaneous wound, the animals were randomized into three groups (10 animals in each group); the untreated group, the group treated with 0.1 ml of Ok Au NPs colloidal solution, and the group treated with Ch Au NPs colloidal solution. The treatment was performed for the wound on 12 consequent days. A digital calliper was used to measure the changes in wound area diameter (mm). For histological examination, all animals were euthanised on the 12th day of the surgery. The wound and the surrounding skin were thoroughly removed for histopathological staining. The samples were fixed with 10% formalin, dehydrated with different graded alcohol concentrations, cleared with xylene, and embedded in paraffin. The sections of 5 *μ*m were prepared with Masson's trichrome (MT) and H&E method and histological changes surveyed by optical microscopy (Olympus).

### 2.7. Statistical Analysis

The data were analyzed by one-way ANOVA using the SPSS v22 software package. *P* < 0.01 was a limit of significance.

## 3. Result and Discussion

### 3.1. UV-Vis

At first, Au NPs synthesis in the solution and their surface plasmon resonance (SPR peaks) and size were confirmed using a UV-Vis spectrophotometer (Perkin-Elmer, Lambda 25) in the range of 200 to 700 nm. Curve (a) in Figure 3 shows the spectrum of okra extract. Curve (b) in Figure 3 shows the spectrum of green synthesized Au NPs (Ok Au NPs) containing a perfectly sharp and strong peak at 538 nm, and there was an increase in intensity till 5 min as a function of time without any shift in the peak wavelength which indicated the presence of Au NPs (∼55 nm). Finally, Curve (c) in Figure 3 shows the spectrum of chemical synthesized Au NPs (Ch Au NPs). The peak at 516 nm demonstrated Au NPs (10 nm) in the solution, Figure 3. The presence of these two sharp bands was attributed to the SPR of Au NPs [36]. The shape and size SPR band may contribute to its development during the generation of Au NPs [37]. This can also be verified by the development of rod-like and spherical Au NPs. The achievement of saturation in the bio-reduction of Au_3_+ may also be involved in this. Generally, there is a positive correlation between the reduction of gold ions to Au NPs and the intensity of the SPR peak. The complete reduction of gold ions to Au NPs is shown by developing a stable dark purple color in the reaction mixture over 5 minutes [38].

### 3.2. FTIR

Spectrum of okra extract in Figure 4(a) shows peaks at 3344 cm^−1^ (O–H stretch), 2926 cm^−1^ (C–H stretch), 1612 cm^−1^ (C = O stretch), 1444 cm^−1^ (C–C stretch), and 1045 cm^−1^ (C–N stretch).  Figure 4(b), which is for green synthesized Au NPs, shows peaks at 34415 cm^−1^ (O–H stretch), 2924 and 2854 cm^−1^ (C–H stretch), 1618 cm^−1^ (C = O stretch), 1458 cm^−1^, 1379 cm^−1^ (C–C stretch), and 1163 cm^−1^ (C–N stretch).  Figure 4(c), for chemical synthesized Au NPs, shows peaks at 3414 cm^−1^ (O–H stretch), 2954 and 2924 cm^−1^ (C–H stretch), 1618 cm^−1^ (C = O stretch), 1458 cm^−1^, 1379 cm^−1^ (C–C stretch), and 1165 cm^−1^ (C–N stretch). As a result, one band at 540 cm^−1^ disappeared and another new band was developed at 476 cm^−1^ (Figure 4(b)) and 474 cm^−1^ (Figure 4(c)) corresponding to N–H groups in proteins and formation of metal Au NPs peaks. FTIR results showed that the extracts containing hydroxyl group as a functional group could bind to and decrease the metal ions to metal nanoparticles, indicating the mechanism for the reduction of gold ions to gold nanoparticles [37].

On the other hand, the FTIR analysis displayed that reducing the nanoparticles by biomolecules present in the aqueous extract of okra could be responsible for binding onto the gold surfaces to make the particles stable.

### 3.3. XRD

The structure of synthesized Ok Au NPs was determined using XRD analysis and X′ Pert Pr instrument acting at the voltage of 40 KV and current of 30 MA with CUK radiation. Diffraction peaks appear at 38.3, 44.44, 64.72, and 77.66 in a 2ɵ range 0–80. These peaks were related to (111), (200), (220), and (311) facets of a face-centred cubic crystal structure (JCPDS no. 004–0784). Therefore, the crystalline structure of prepared Au NPs with okra extract was confirmed (Figure 5). We have calculated the average size of Au NPs according to the XRD data and Scherrer Equation, which was 77.58 nm.

### 3.4. TEM

The size and shape of Ok Au NPs were determined by transmission electron microscopy (TEM). TEM images obtained from the Zeiss-EM10C-100 KV instrument are shown in Figure 6 with different resolutions. It demonstrated that gold nanoparticles have almost a spherical morphology without agglomeration. Our result was in agreement with the shape of SPR bands centred at 450 nm of colloid. The original TEM, shown in Figure 6, was digitally processed using MATLAB [39]. The method used to process the image was based on local thresholding, which helps us in particle counting, mean diameter measurement, and obtaining the size distribution diagram. The outputs of digital image processing are shown in Figures 6 and 6(c). The outputs confirmed the presence of 586 NPs with a mean diameter of 75 nm.

### 3.5. Antioxidant Activity

Recently, the application of medicinal plants with antioxidant and anti-inflammatory activity has increased. Antioxidant compounds reduce the free radicals in the wound area and enhance wound healing [40]. Metal nanoparticles have efficient antioxidant properties against DPPH free radical scavenging [41]. By reducing the free radicals in the wound area, the antioxidant compounds help to heal the wound. Other studies have shown that medicinal plants enriched with antioxidant and anti-inflammatory compounds improve wound healing [7, 40]. DPPH radical scavenging effect of Ok Au NPs and Ch Au NPs was compared to Vit C in five different concentrations (Figure 7). It has been suggested that the free radical scavenging activity of Ch Au NPs and Ok Au NPs is enhanced with an increase in the concentration of Au NPs in the range of 20–100 µg/ml. Our results showed that Ch Au NPs, Ok Au NPs, and vitamin C have antioxidant activities. However, in this study, the Au NPs had a suitable wound healing activity (Figure 7).

### 3.6. Cytotoxicity Survey

The cytotoxicity potentials of Au NPs were measured in different concentrations (0, 7.5, 15, 30, 60, 100, 150, and 200 *μ*g/mL) against HDF cell line using MTT assay for 24 h (Figure 8). Furthermore, the absorbance rate was measured at 570 nm, which displayed excellent viability on a normal HDF cell line at concentrations up to 200 *μ*g/ml for Au NPs. In addition, we observe that Au NPs did not cause significant cytotoxicity in the range of used concentrations for MTT assay (Figure 7).

In line with our study, Hamelian et al. reported that when plant compounds are mixed with gold salts, their cytotoxicity is eliminated [41]. Bartczark et al. studied the cytotoxicity of hollow gold spheres, gold nanospheres, and core/shell silica/gold nanocrystals against endothelial cells and discovered noncytotoxic effects [42].

### 3.7. Antimicrobial Activity

MIC values for *Escherichia coli*, *Klebsiella pneumoniae*, *Staphylococcus aureus*, and *Bacillus subtilis* are 10.75, 13.80, 10.83, 9.90 *μ*g/mL and 9.57, 10.58, 10.21, 8.95 for Ok Au NPs and Ch Au NPs, respectively. Still, the values of MBC are 22.01, 21.75, 21.65, 19.80 *μ*g/mL and 19.35, 20.50, 20.25, 17.45 *μ*g/mL for Ok Au NPs and Ch Au NPs (Table 1). As the results of Table 1 showed, synthesized Ok Au NPs and Ch Au NPs have prevented the growth of indication bacteria. Increasing the concentration of Au NPs enlarged the inhibition zone.MIC: minimal inhibitory concentration; MBC: minimal bactericidal concentration; C: concentration; ZOI: zone of inhibition.

Nanoparticles have a significant antibacterial effect, and this effect is intensified by increasing the concentration of nanoparticles. The mechanism of resistance to antibiotics does not lead to resistance to antibacterial compounds in nanoparticles. Regarding the mechanism of antibacterial properties of nanoparticles, it was stated that nanoparticle ions react with live bacterial enzymes and inactivate them. Also, as a catalyst, it converts oxygen to activated oxygen (including hydroxyl radicals). This reaction is carried out by light energy in air or H_2_O and only at the polar surfaces; therefore, reactive oxygen inhibits the growth of bacteria [43]. It should be noted that for the direct contact of nanoparticles with bacteria, their size should be between 1 and 10 nm. In this study, the average size of nanoparticles was 40 nm, which had the greatest antibacterial effect. In the presence of nanoparticles, microorganisms lose their ability to replicate, and cell proteins are inactivated [44]. Therefore, bacterial resistance to chemical antibiotics does not cross-react with these nanoparticles. This is a point of hope for using antibacterial compounds of these nanoparticles in the treatment of infections, especially infections with antibiotic-resistant bacteria [45].

### 3.8. In Vivo Study

This study showed an enhanced percentage of wound closure and diameter of the wound area (Figures 9 and 10). As illustrated in Figures 9 and 10, treatment with Ok Au NPs improved the size of the wound area diameter and the percentage of wound closure, which is in agreement with previous reports [38]. Percentage of wound closure = (1 − (wound area)/(original wound area) × 100).

#### 3.8.1. Histopathology

To evaluate the histological changes of the skin, hematoxylin and eosin (H&E) and Masson's trichrome (MT) staining were performed in health and wound tissue samples. In healthy skin, the stratum of the *epidermis*, dermis (connective tissue with skin appendages), and hypodermis are observed (Figure 11). A wide necrotic tissue was observed on the surface part of the wound in the untreated group due to the injury. In the necrotic tissue, there was the secretion of inflammatory cells with blood cells. In this tissue, collagen fibers in the extracellular matrix were discrete and irregular in the MT section. In the group receiving Ok Au NPs and the Ch Au NPs, the accumulation of inflammatory cells and the dispersion of collagen fibers were observed in the formed epithelial tissue (Figure 12). In groups treated with the Au NPs, the epithelium was formed on a large scale. In addition, there were organized collagen fibers in the dermis and blood vessels; also, aggregation of natural cells was observed at the wound area. In this group, the MT section showed a large amount of collagen. In general, in the treated groups, the formed epithelial tissue was thicker than normal rats, and skin appendages were not observed (Figure 12). In agreement with the findings mentioned above, Au NPs reduce histopathological changes in the wound healing condition possibly through different mechanisms such as angiogenesis pathway, alteration in the membrane potential and triggering the optimum intracellular ROS, and enzyme ATP synthase [38].

## 4. Conclusions

This study indicated that synthesizing Au NPs using aqueous okra extract is an ecofriendly, simple, and useful method. UV/Vi*s* spectroscopy, FTIR, XRD, and TEM techniques were used to characterize the Ok Au NPs synthesized. Furthermore, the favorable antibacterial and antioxidant activities of the green synthesis of Au NPs could be a safe and effective adjuvant for wound healing. Therefore, Ok Au NPs may be ideal candidates for future studies discovering their use in therapeutic and pharmaceutical applications.

## Figures and Tables

**Figure 1:** Graphical abstract of green/chemical synthesis of Au NPs.

**Figure 2:** Images of the culture plates seeded with *Escherichia coli* (ATCC 11775), *Klebsiella pneumoniae* ATCC 13883, *Staphylococcus aureus* ATCC 33591, and *Bacillus subtilis* ATCC 605 so that the inhibition zone created by the samples can be observed.

**Figure 3:** UV-Vis absorption spectra of okra extract (a), Au NPs synthesized from okra (Ok Au NPs) (b), and a solution containing Ch Au NPs (chemical synthesis) (c).

**Figure 4:** FTIR spectra of (a) okra extract, (b) green synthesized Au NPs (Ok Au NPs), and (c) chemical synthesized Au NPs (Ch Au NPs).

**Figure 5:** XRD spectrum showing peaks corresponding to the diffraction from (111), (200), (220), and (311) planes of fcc lattice of Ok Au NPs.

**Figure 6:** (a) The original TEM image, (b) particles which were detected by local thresholding, and (c) particle size distribution diagram obtained from the analysis of the TEM image.

**Figure 7:** Antioxidant activity of Ch Au NPs, Ok Au NPs, and Vit C.

**Figure 8:** Cell viability of Ch Au NPs and Ok Au NPs on HDF cells after 24 h incubation at different concentrations (0, 7.5,15, 30, 60, 100, 150, and 200 *μ*g/ml).

**Figure 9:** Wound status in the experimental groups.

**Figure 10:** The percentage of wound closure for the control group, group Ch Au NPs, and group Ok Au NPs (mean ± SEM, *n* = 5). *P* < 0.05 is a significant level compared to the control group.

**Figure 11:** Histopathological images of the skin from the different groups with hematoxylin and eosin (H&E) and Masson′s trichrome (MT) staining: healthy group showing normal histological structure and wound group in which intense skin damage can be observed.

**Figure 12:** Histopathological images of the skin from the different groups with hematoxylin and eosin (H&E) and Masson's trichrome (MT) staining: the wound groups treated with the Ok Au NPs and the Ch Au NPs in which there was an improvement in the tissue structure.

**Table 1:** Antibacterial characteristics of Au NPs.

microorganism	Test extracts	MIC (*μ*g/mL)	MBC (*μ*g/mL)	ZOI chloramphenicol and tetracycline (mg/mL)
*Escherichia coli*	Ok Au NPs	10.75	22.01	0.35
	Ch Au NPs	9.57	19.35	0.35

*Klebsiella pneumoniae*	Ok Au NPs Ch Au NPs	13.80 10.58	21.75 20.50	0.35

*Staphylococcus aureus*	Ok Au NPs	10.83	21.65	0.35
	Ch Au NPs	10.21	20.25	0.35

*Bacillus subtilis*	Ok Au NPs	9.90	19.80	0.35
	Ch Au NPs	8.95	17.45	0.35

## Data Availability

Raw data associated with this study are available from the authors upon a reasonable request.
